RETRACTED

# Iron Supplementation Decreases Severity of Allergic Inflammation in Murine Lung

**DOI:** 10.1371/journal.pone.0045667

**Published:** 2012-09-20

**Authors:** Laura P. Hale, Erin Potts Kant, Paula K. Greer, W. Michael Foster

**Affiliations:** 1 Department of Pathology, Duke University Medical Center, Durham, North Carolina, United States of America; 2 Department of Medicine/Division of Allergy, Pulmonary, and Critical Care Medicine, Duke University Medical Center, Durham, North Carolina, United States of America; 3 Human Vaccine Institute, Duke University Medical Center, Durham, North Carolina, United States of America; French National Centre for Scientific Research, France

## Abstract

The incidence and severity of allergic asthma have increased over the last century, particularly in the United States and other developed countries. This time frame was characterized by marked environmental changes, including enhanced hygiene, decreased pathogen exposure, increased exposure to inhaled pollutants, and changes in diet. Although iron is well-known to participate in critical biologic processes such as oxygen transport, energy generation, and host defense, iron deficiency remains common in the United States and world-wide. The purpose of these studies was to determine how dietary iron supplementation affected the severity of allergic inflammation in the lungs, using a classic model of IgE-mediated allergy in mice. Results showed that mice fed an iron-supplemented diet had markedly decreased allergen-induced airway hyperreactivity, eosinophil infiltration, and production of pro-inflammatory cytokines, compared with control mice on an unsupplemented diet that generated mild iron deficiency but not anemia. *In vitro*, iron supplementation decreased mast cell granule content, IgE-triggered degranulation, and production of pro-inflammatory cytokines post-degranulation. Taken together, these studies show that iron supplementation can decrease the severity of allergic inflammation in the lung, potentially via multiple mechanisms that affect mast cell activity. Further studies are indicated to determine the potential of iron supplementation to modulate the clinical severity of allergic diseases in humans.

## Introduction

Under normal conditions, the immune system responds to common ingested or inhaled antigens by inducing a state of specific non-responsiveness called tolerance. Allergy develops when antigen-presenting cells process these otherwise innocuous antigens and present them to T cells in a cytokine milieu that promotes B cell production of allergen-specific IgE. When allergen-specific IgE bound to mast cell Fc receptors is cross-linked by allergen, the mast cells release pre-formed granules containing histamine, TNF, IL-8 and other inflammatory mediators. Mast cell degranulation thus induces a cascade that results in infiltration by immune cells and and stimulates *de novo* production of additional inflammatory mediators. Inflammation may be localized to the site of exposure (e.g. respiratory or gastrointestinal tracts) or may become systemic, resulting in life-threatening episodes of anaphylaxis.

RETRACTED

Asthma is a chronic inflammatory disease of the airways associated with airway hyperresponsiveness that often occurs in allergic patients. Despite an intensive research effort to identify mechanisms central to the diathesis of inflammatory airway disease, control factors remain unclear [1]. The incidence of asthma is increasing and affects 300 million people worldwide, including 23 million in the US, where it leads to 5,000 deaths annually [2]. Current treatments that decrease the severity of airway obstruction include bronchodilators and corticosteroids, but these fail to address any underlying allergic reactions. Methods to decrease the severity of allergic reactions include IgE depletion using anti-IgE monoclonal antibodies, induction of IgG blocking antibodies by allergen immunotherapy, and blocking downstream effects of mast cell degranulation using antihistamines or corticosteroids. Controlled oral exposures to allergens have in some cases allowed subjects to develop tolerance, although the mechanisms involved are still under active investigation. However, many asthma patients go on to develop treatment-resistance and disease progression despite optimized treatments, [3], [4]. Identification of additional therapies that could prevent or decrease the severity of allergic reactions would provide a major improvement in clinical care of patients with allergen-triggered asthma.

Iron status is well-known to affect the ability to oxygenate tissues and generate energy, but how iron affects immune and non-immune-triggered inflammatory processes is less clear. We recently identified iron deficiency as a trigger for increased mast cell activation that was associated with mast cell-dependent hair loss in IL-10-deficient (*Il10* ^−/−^) mouse pups [5]. The effects of iron status on mast cell reactivity in classic mast cell-mediated diseases such as allergy have not been reported previously. These studies were designed to test the hypothesis that iron supplementation could beneficially decrease the severity of allergic disease by decreasing mast cell activation, using a classic model of IgE-mediated allergic asthma in mice.

## Methods

### Ethics Statement

All animal studies were approved (protocol numbers A151-09-05 and A190-09-07) by the Institutional Animal Care and Use Committee of Duke University, an institution accredited by the Association for Assessment and Accreditation of Laboratory Animal Care (AAALAC), International. Suffering was minimized by providing anesthesia for all procedures (the Flexivent measurements) with the potential to cause pain and/or distress.

RETRACTED

### Animal Studies

Breeding pairs of C57BL/6 wild type (WT) and mast cell-deficient *Kit* ^W-sh^/*Kit* ^W-sh^ (*Sash*) mice (strain name  =  *B6.Cg-Kit^W-sh^/HNihrJaeBsmJ*; stock #005051) [6], [7] were obtained from Jackson Laboratories (Bar Harbor, ME). Experimental mice were placed on AIN-93G- based custom diets containing 8 or 200 ppm iron at 3–4 weeks of age. Four weeks later, mice were sensitized to ovalbumin (OVA) by intraperitoneal immunization with 20 µg OVA +2 mg alum on day 0 and 10 µg OVA +1 mg alum on day 7, then challenged by a 20 min exposure to aerosolized 1% OVA or saline on days 14, 15, 16. On day 17, mice were anesthetized and total airway resistance in response to nebulized methacholine was measured as described [8]. Only male mice were used, since males and females differ in both iron homeostasis [9] and susceptibility to asthma [10].

Erythropoiesis was determined by a complete blood count (CBC). Non-heme iron stores in liver and spleen were determined colorimetrically [11]. Serum iron was measured using a commercially available kit (Thermo Scientific, Middletown, VA). Hepcidin transcript levels were determined by real-time reverse transcriptase PCR of liver tissue [12] and expressed as 2^−ΔΔCt^, based on the threshold cycle (Ct) for hepcidin compared to *β*-actin, OVA-specific IgG was quantitated by antibody capture enzyme immunoassay on immobilized OVA [13]. OVA-specific IgE was measured by antibody capture on immobilized anti-IgE, followed by binding and quantitation of biotinylated OVA via a standard curve with known concentrations of anti-OVA IgE (clone PMP68; AbD Serotec, Raleigh, NC).

Bronchoalveolar lavage (BAL) samples were obtained following euthanasia. Cytokines were quantitated by a Luminex bead-based multiplex fluorescent immunoassay (BioRad). Mucous (goblet cell) metaplasia was evaluated using periodic acid-Schiff (PAS)-stained lung sections. For analysis of *Muc5AC* transcripts, total RNA was extracted from ∼30 mg lung tissue. cDNA was synthesized and real-time PCR analyses were performed using SYBR green fluorescence and specific primers [14]. Relative levels of *Muc5AC* transcripts were expressed as 2^−ΔΔCt^ versus *β*-actin.

### *In vitro* Studies of Mast Cell Activation

Primary bone marrow-derived mast cells (BMMC) were derived as described [15] using 10% fetal bovine serum with an iron content of 193 µg/dL (79% transferrin saturation). For degranulation assays, sensitized BMMC were incubated with ± iron for 30 min prior to activation. RBL-2H3 mast cells (American Type Culture Collection; Manassas, VA) were cultured for 20 hrs in media containing 1 µg/ml IgE and 10% calf serum with low (25 µg/dL Fe; 5% transferrin saturation), medium (low supplemented to 642 µg/dL Fe; 83% transferrin saturation), or high iron content (medium serum supplemented to 1402 µg/dL Fe with 50 µM FeSO_4_). Degranulation was triggered by cross-linking with goat anti-mouse IgE antibody in serum-free Tyrode’s buffer. Percent degranulation was determined using a colorimetric substrate assay for β-hexoseaminidase as described [16]. Total granule content was determined following lysis with Triton X-100. Viability after degranulation was monitored using a tetrazolium-based colorimetric assay.

RETRACTED

## Results

### Iron Supplementation Decreases the Severity of Allergic Asthma

At 3–4 weeks of age, wild type (WT) C57BL/6 male mice were placed either on an unsupplemented diet containing 8 ppm iron or a matched diet supplemented to contain 200 ppm iron. The recommended daily amount of iron for mice is 35 ppm [17] and 200 ppm is a level commonly used for iron-supplemented rodent diets. Beginning at 8–9 weeks of age, all mice were sensitized to ovalbumin (OVA) then challenged x 3 with aerosolized OVA or saline and airway resistance was determined following methacholine challenge. OVA-challenged mice that consumed the unsupplemented (8 ppm iron) diet showed large methacholine-induced increases in airway resistance compared with saline-challenged mice (Figure 1A). These changes in airway resistance were markedly attenuated (∼30% reduction) in OVA-challenged mice on the iron-supplemented (200 ppm) diet (Figure 1A; p≤0.0005). Allergen triggering induced marked infiltration of inflammatory cells into bronchoalveolar spaces of unsupplemented mice (mean ± SEM = 202,408 total cells/ml), the majority of which were eosinophils. This cellular infiltration was also markedly attenuated by iron supplementation (Figure 1B). Specifically, the eosinophils present in bronchoalveolar spaces decreased from 192,679±12,608 eosinophils/ml BAL fluid in OVA-challenged unsupplemented mice (95% of total cells; n = 5 mice) to 93,224±13,770 eosinophils/ml in OVA-challenged iron-supplemented mice (85% of total cells; n = 5 mice), a decrease of ∼50%. Production of a variety of proinflammatory cytokines and chemokines within pulmonary tissue were also significantly decreased by iron supplementation. These included IL-1β, IL-3, IL-4, IL-5, Il-6, IL-9, IL-10, IL-12(p40), IL-13, IL-17, IFN-γ, KC, GM-CSF, and MIP1α (Figure 2A–C).

RETRACTED

**Figure 1:** Iron supplementation decreases severity of allergic asthma. WT and mast cell-deficient *Sash* mice on the indicated diets were sensitized to OVA then challenged with OVA or saline. **A**. Airway resistance (measured in units of cm H_2_O/ml/sec) in response to methacholine was significantly decreased following allergen challenge for mice that received iron supplementation (*indicates p≤0.0005). **B**. Iron supplementation decreased infiltration of eosinophils into bronchoalveolar spaces (decrease of 52%; *indicates p = 0.0007).

**Figure 2:** Effects of iron supplementation on allergen-induced cytokine secretion into bronchoalveolar spaces. Cytokine and chemokines present in bronchoalveolar lavage (BAL) fluid obtained from OVA-sensitized mice 24 hrs following the 3d challenge with aerosolized antigen or saline were markedly increased in unsupplemented compared with iron-supplemented mice (*indicate p<0.01). The percentage increase ranged from 25–35% for IL-1β, IL-5, IL-6, and IL-13 to 170% for IL-17.

As typically seen in allergic asthma [18], allergen challenge also induced mucous metaplasia, with increased numbers of goblet cells present in the large airways of OVA-challenged mice from both diet groups (Figure 3A–D). Mucus production increased following allergen challenge as measured by qPCR for Muc5AC mRNA, but was not affected by iron supplementation (Figure 3E).

**Figure 3:** Iron supplementation does not affect mucus production. Periodic acid-Schiff (PAS)-stained formalin-fixed, paraffin-embedded lung sections show allergen-induced goblet cell differentiation in the large airways of mice on both 8 ppm (**A**  =  saline-challenged, **B**  =  OVA-challenged) and 200 ppm diets (**C**  =  saline-challenged, **D**  =  OVA-challenged). Expression of Muc5AC mRNA in the lungs was similar for both diet groups (**E**).

### Effect of the Unsupplemented Diet on Iron Status and Allergic Sensitization

Total body iron content is reflected by iron present in red blood cells, serum, and stored within tissues. When dietary iron is limited, its absorption is enhanced by inhibition of the iron regulatory hormone hepcidin and additional iron is mobilized from tissue stores to maintain normal levels of serum iron and hematopoiesis. Once tissue iron stores are depleted, iron deficiency anemia will result if iron intake remains insufficient to meet daily iron needs. Tissue iron content is thus the most sensitive measure of body iron status. Hepcidin production was determined in allergen-sensitized but saline-challenged mice to avoid confounding due to effects of inflammation. At the time of allergen challenge, hemoglobin and hematocrit were slightly decreased for mice on the 8 ppm iron diet compared with the iron-supplemented diet (Table 1), but remained in the normal range. Tissue analysis revealed that these mice had markedly decreased levels of iron stored in liver and spleen. The low ratios of hepcidin:actin mRNA (Table 1) measured in unsupplemented mice are consistent with the expected ongoing release of stored and newly absorbed iron into the systemic circulation, based on their mild to moderate iron deficiency without anemia. Interestingly, serum iron levels were slightly elevated in unsupplemented mice, most likely reflecting extensive mobilization of body iron stores (Table 1). Thus, although the mice on the unsupplemented diet had deficient iron stores, their degree of iron deficiency was not sufficient to result in anemia. The higher levels of hepcidin transcripts seen in the mice on the iron-supplemented diet is consistent with their higher total body iron stores and therefore a decreased need for release of recently absorbed or stored iron.

RETRACTED

**Table 1:** Iron Status of Mice Studied.**

	UnsupplementedDiet (8 ppm iron)	SupplementedDiet (200 ppm)
RBC (M/µL)	10.2±0.3	10.1±0.3
Hgb (g/dL)	14.6±0.5	15.7±0.3*
Hct (%)	46±2	50±1
MCV (fL)	44.7±1.9	49.7±0.9*
Serum iron (µg/dL)	193±8	174±9*
Liver iron (µg/g wet tissue)	16±2	88±3
Spleen iron (µg/g wet tissue)	45±9	270±19
Hepcidin:actin mRNA (liver)	0.05 (0.02–0.12)	1.82* (1.50–2.22)

* indicates p≤0.05 for comparisons of unsupplemented vs. iron-supplemented diets.

** Data shown are mean ± SEM for 6 mice/diet group for red blood cells (RBC), hemoglobin (Hgb), hematocrit (Hct), and mean cellular volume (MCV). The numbers of mice studied for serum and tissue iron ranged from 10–25 per group. Hepcidin measurements are given as the geometric mean (upper - lower confidence interval) for 10 allergen-sensitized, saline-challenged mice/group.

Similar levels of OVA-specific antibodies were present in the serum of mice on the unsupplemented diet (186±7 µg/ml OVA-specific IgG and 122±15 ng/ml OVA-specific IgE; n = 25) compared with mice on the iron-supplemented diet (173±7 µg/ml OVA-specific IgG and 123±20 ng/ml OVA-specific IgE; n = 12). Thus, under the conditions used for this study, iron supplementation did not affect asthma severity through effects on allergic sensitization.

Although it has been reported that the OVA-alum model of asthma is not necessarily mast cell-dependent [19], this has been refuted by others [20]–[22]. We found that allergen-induced airway responses were minimal in mast cell-deficient Kit^W-sh^/Kit^W-sh^ (*Sash*) mice that were sensitized and challenged with OVA (Figure 1A). This indicated that, under the experimental conditions used for this study, contributions of non-mast cells to the changes in airway resistance in this model were small. Thus, the differences in airway resistance measured primarily resulted from allergen-triggered activation of mast cells.

RETRACTED

### Iron Supplementation Decreases Mast Cell Activation *in vitro*

To directly assess the effects of iron supplementation on mast cells, IgE-sensitized primary bone marrow-derived murine mast cells (BMMC) were incubated in Tyrode’s buffer, with and without addition of 100 µM Fe^2+^ for 30 min prior to activation via IgE cross-linking. Iron supplementation had no effect on spontaneous degranulation, but decreased IgE-mediated degranulation by 30% (p = 0.01; Figure 4A). Following degranulation, BMMC were cultured for 18 hrs in their standard growth media and selected cytokines and chemokines were measured by multiplex fluorescent immunoassay. Production of TNF, MCP-1, and IL-6 by IgE-activated mast cells was markedly decreased by iron supplementation, with reductions of 94%, 29%, and 27%, respectively (Figure 4B). Baseline levels of IL-1β, IL-4, IL-10, IFN-γ, KC, and MIP-1α produced by BMMC were extremely low at this time point and were not affected by IgE-mediated degranulation or by iron supplementation. Additional studies using the RBL-2H3 rat mast cell line showed that iron supplementation also decreased mast cell granule content, measured both by total cellular content of the granule-associated enzyme β-hexoseaminidase content and by flow cytometric detection of cytoplasmic granularity (Figure 4C–E).

**Figure 4:** Effects of iron supplementation on IgE-mediated mast cell degranulation, cytokine production, and total granule content. **A**. Supplementation with iron decreased degranulation of primary BMMC by 30% (*indicates p = 0.01). Data shown is the mean ± SEM of 4 experiments. **B, C**. In duplicate experiments, iron supplementation decreased mast cell production of TNF, MCP-1, and IL-6 by 94%, 29%, and 27%, respectively. An MTS assay confirmed continued viability of the BMMC (not shown). **D, E**. RBL-2H3 mast cells showed a dose-dependent reduction in total granule contents per cell with iron supplementation, as indicated by β-hexoseaminidase activity following lysis with Triton X-100 (panel D) and flow cytometric analysis of side scatter (panel E). Data shown represents the mean ± SEM of 3 − 4 independent experiments, each conducted in triplicate. *indicates p≤0.02.

## Discussion

These studies show that dietary iron supplementation decreased the severity of allergic asthma in wild type mice, as measured by significant decreases in infiltration of eosinophils and secretion of proinflammatory cytokines and chemokines into bronchoalveolar spaces, confirming in part similar results recently reported by Maazi *et al* [23]. In addition, we made the novel observation using a direct measure of airflow resistance that supplementation attenuates the acute development of airway hyperresponsiveness in the common ovalbumin model of allergic asthma. In our studies, the benefits of iron supplementation were observed in mice with levels of iron deficiency that would be classified clinically as mild, since body iron stores were decreased but not serum iron levels or hematopoiesis. *In vitro* studies showed that iron supplementation affected mast cell activity via multiple mechanisms that included decreased mast cell granule content, decreased IgE-mediated degranulation, and decreased production of pro-inflammatory cytokines and chemokines following degranulation.

RETRACTED

Few studies regarding potential effects of iron on mast cell activity have been reported previously. Incubation of mast cells with media containing serum or the iron-containing protein transferrin was previously described to inhibit mast cell degranulation [24]. Conversely, exposure to iron chelators has been shown to activate primary human mast cells [25], [26], rat peritoneal mast cells [25], [27], and a human mast cell line [28]. Our *in vitro* studies confirm that iron supplementation also has direct inhibitory effects on mast cell activation.

Our *in vivo* studies also clearly show that iron supplementation can decrease the severity of inflammation in an *in vivo* model of allergic asthma in mice with mild iron deficiency. It is tempting to speculate that these effects are directly due to effects of iron on mast cells, particularly in light of our data that mast cells are required for the differences in airway resistance seen in iron-supplemented vs. unsupplemented mice following allergen challenge (Figure 1A). However, these results do not rule out potential significant contributions by other cell types to decrease airway responses upon iron supplementation. Although iron supplementation was shown to decrease total mast cell granule content as well as IgE-triggered mast cell degranulation and production of pro-inflammatory cytokines and chemokines post-degranulation, studies that allow manipulation of iron levels within specific cell types, including mast cells, will likely be required to further define the cell types involved as well as the precise mechanisms by which iron regulates these processes.

Iron supplementation reduced production of a number of pro-inflammatory cytokines and chemokines following respiratory exposure to aerosolized allergen (Figure 2). Each of these agents has previously been shown to contribute to the pathogenesis of asthma [29], [30], and demonstration of these important biologically relevant mechanisms for decreased airway hypperreactivity and inflammation adds strength to the study. In particular, IL-9 has been shown to be critical in the pathogenesis of bronchial hyperresponsiveness. Our finding that IL-17 production is also decreased by iron supplementation is also of particular interest, given recent data suggesting that IL-17-producing Th17 cells can also play a pathogenic role in allergic asthma [30].

RETRACTED

In addition to effects on allergen-induced pathways of inflammation, it is also possible that iron may affect mast cell activity directly via its redox properties. Cho *et al* recently showed that stimulation of mast cells through FcεRI induced the production of intracellular reactive oxygen species that act as second messengers in a signal transduction pathway leading to degranulation and cytokine synthesis [31]. Iron is a well-known quencher of free radicals and can be readily oxidized or reduced under conditions present within cells. But at present, neither the source of the reactive oxygen species generated in response to Ag stimulation nor the pathway by which they are generated in Ag-stimulated mast cells is clearly understood. Iron homeostasis in mast cells is also poorly understood. Thus, additional studies will be required to determine the potential contribution of these pathways to asthma severity.

Although mice with decreased iron stores had more severe inflammation in this model of allergic asthma, the iron-dependent changes in immune cell reactivity that we observed may potentially be beneficial to host defense. Mast cells are best known for their pathogenic role in allergy and asthma. However, their immediate release of pre-stored TNF upon degranulation stimulates a rapid influx of neutrophils that is critical for control of bacterial infections. Mice deficient in mast cells are thus highly susceptible to fatal infections with enteric bacteria [32], [33]. TNF released by mast cells is also critical for inducing lymph node changes that stimulate the development of antigen-specific immune responses [34]. Following degranulation, mast cells continue to secrete cytokines that further stimulate the inflammatory response. Inflammation induces the peptide hormone hepcidin, which decreases bioavailable iron to additionally limit bacterial growth [35]. Thus, based on current understanding of these pathways, enhanced mast cell activation due to decreased iron could be beneficial to enhance host antibacterial defenses, but enhanced mast cell activation is detrimental in allergy.

RETRACTED

The potential to decrease the severity of allergic reactions by normalizing iron status has major implications for public health, since correction of iron deficiency is simple, safe, and inexpensive and is medically desirable for a variety of reasons. Iron deficiency is the most common nutritional deficiency in humans world-wide [36]. The Centers for Disease Control and Prevention estimates that, in the United States, 7% of children 1–2 yrs of age, 12% of females from ages 12–49, and 2% of males from ages 16–69 have severe iron deficiency with or without anemia [9]. In a setting of iron sufficiency, the iron-regulatory hormone hepcidin maintains body iron homeostasis by decreasing dietary iron absorption and preventing release of stored iron into the bloodstream [37]. Since production of hepcidin is also up-regulated by inflammation [38], the inflammatory sequelae of allergic reactions would be predicted to exacerbate any dietary iron deficiency by further decreasing iron absorption and release.

It is important to note that, although the unsupplemented mice in our study had significantly decreased iron stores, the large increases in airway resistance occurred while hematologic parameters (e.g. Hgb, Hct) remained within the normal range. Humans with a similar degree of iron deficiency would not typically be classified as being iron-deficient based on a complete blood count. Measurement of iron stores in humans currently requires expensive (e.g. magnetic resonance imaging [39]) or invasive testing (e.g. bone marrow biopsy). Identification of alternative blood-based biomarkers of iron status that can accurately predict mast cell reactivity will facilitate follow-up studies to determine the potential of iron supplementation to modulate the clinical severity of allergic diseases in humans.
